This article has been retracted.

# Application of PDCA Process Management in Day Operation Ward and the Influence of Nursing Quality and Safety

**DOI:** 10.1155/2022/8169963

**Published:** 2022-03-07

**Authors:** Huan Ma, Juan Cao, Meng Li

**Affiliations:** Day Surgery Center, The Central Hospital of Wuhan, Tongji Medical College, Huazhong University of Science and Technology, Wuhan 430014, China

## Abstract

**Objective:**

To survey the application of PDCA (plan, do, check, and action) process management in day operation ward and the influence of nursing quality and safety.

**Methods:**

The routine nursing management was carried out in our hospital from March 2019 to March 2020, which was set as the control group (*N* = 20), and the PDCA process management was implemented from March 2020 to March 2021 as the research group (*N* = 20). Twenty nurses and patients were selected as subjects in two periods of time. The nursing quality, the score of individual quality control examination in clinical department, the nursing quality of operating room, the incidence of adverse events and nursing errors, the number of problems existing in the quality management of nursing documents, and the score of nursing satisfaction were accessed.

**Results:**

In the comparison of nursing quality, the nursing safety, specialty quality, and nursing norms of the study group were higher compared to the control (*P* < 0.05). In terms of the scores of individual quality control examination in clinical departments, the scores of ward management, rescue, therapeutic articles, drug management, first-level nursing, nursing documents, and head nurses in the study group were greater compared to the control (*P* < 0.05). In terms of the operating room nursing quality score, the instrument management, instrument preparation, nurses' cooperation skills, disinfection and isolation quality, and the total score of the study group were above the control (*P* < 0.05). In terms of the incidence of operative adverse events and nursing errors, the incidence of nosocomial infection, iatrogenic injury, information check error, equipment failure, violation of operation regulations, ECG monitoring error, infusion operation error, and medication error in the study group was lower compared to the control (*P* < 0.05). According to the comparison of the number of problems existing in the quality management of nursing documents, the number of problems in temperature sheet, medical order, evaluation sheet, nursing record, and other nursing documents in the study group was lower than the control (*P* < 0.05). The scores of nursing communication, professional technology, nursing service attitude, nursing environment, and knowledge education in the study group were higher in contrast to the control (*P* < 0.05).

**Conclusion:**

The application of PDCA management can effectively enhance the nursing quality and safety of the day operation ward, further facilitate the quality of hospital nursing work, and improve patient satisfaction, which exert great potential, and application value in the management of day ward in the future.

## 1. Introduction

The operating room is not only the key management department of the hospital but also an important place for patients to receive surgical treatment. To a certain extent, the quality of nursing management of the operating room is an important reflection of the medical quality of the hospital, so improving the quality of nursing management of the operating room is beneficial to improve the level of hospital management. Owing to the particularity of nursing in operating room, the current nursing management in operating room is mainly routine management. Although this qualitative method can evaluate the working status and nursing quality of nurses, it has subjective and one-sided restrictions, which will lead to poor management effect. In the long run, it may have an impact on the enthusiasm of nurses, resulting in low work efficiency in the operating room and then affect the satisfaction of patients [1, 2]. In view of these clinical problems, some scholars have put forward the theory of PDCA (plan, do, check, and action) cycle management [3]. With the continuous penetration and influence of the concept of PDCA cycle in the nursing field in China, many nursing researchers in China have applied this theory to the management of nursing quality and achieved good results, but there lacks empirical research on the application of it in the day operation ward [4]. The PDCA theory was used to optimize the nursing quality management process in the day operation ward. The key to the implementation and operation lies in the comprehensive mobilization, the mastery of the whole staff, and the whole process management in all aspects of nursing quality management. Studies have proved that the performance of PDCA theory in nursing work can really put nursing work into practice, improve the connotation of nursing quality service, and improve nursing quality continuously and steadily, so as to improve hospital medical quality [5]. Outpatient surgery is basically a small operation, but at present, due to the large flow of patients and the shortage of nurses in the nursing management of the day operating room, the work is confused and the prevention consciousness is weak, which leads to the poor quality of nursing work in the day operating room [6]. In view of this, in this study, to explore the performance of PDCA process management in the day operation ward and the impact of nursing quality and safety, the research results are reported as follows.

## 2. Patients and Methods

### 2.1. Clinical Information

The routine nursing management was conducted in our hospital from March 2019 to March 2020 (*N* = 20), which was set as the control group, and the PDCA process management was implemented from March 2020 to March 2021 as the research group (*N* = 20). Twenty nurses and patients were selected as subjects in two periods of time. Of the control, the age of nurses was 20-54 years old, with (31.65 ± 1.44) average years old, including 1 male and 19 female, with an average age of (45.67 ± 3.64) years (15-83 years), including 12 males and 8 females. Of the study, the age of nurses was 20-54 years old, with an average of (31.56 ± 1.68) years, including 1 male and 19 female, with an average age of (45.68 ± 3.55) years (13-83 years), including 11 males and 9 females. The general data of nurses and patients of the two were not statistically significant. The study was approved by the Medical Ethics Committee of our hospital.

### 2.2. Nursing Administration

The patient of the control group underwent routine nursing management of the department, and the study group used PDCA process management on the basis of the control group. The specific measures were as follows: (1) stage P (planning stage): a nursing quality management committee was set up to carry out work under the leadership of the hospital quality management committee. The chairman was the dean in charge of nursing work, the vice-chairman was the director of the nursing department, and the members were departmental leaders and committee secretaries. Set up the quality management framework of quality management leading group, quality control team leader, head nurse, and nurse. The head of the quality control team is headed by the director of the nursing department or the head nurse of the major department, and the team member is composed of the head nurse. Meanwhile, all quality control team leaders and team members are required to make hospital nursing quality assessment plans from five aspects of nursing quality evaluation standards: ward management, rescue and treatment materials management, special nursing level basic nursing management, nursing document management, and head nurse management. In order to realize the virtuous circle of assessment, introduce the incentive competition mechanism, formulate the nursing quality competition activity plan, and formulate the whole staff training plan at the implementation level. (2) Stage D (implementation stage): training is carried out according to the plan for decision-making and implementation. Aiming at the decision-making level: organize the members of the quality management leading group to learn the relevant knowledge of total quality management and PDCA management and require to write a relevant summary, and the leaders of each quality control team together with the team members should carefully study the detailed explanation of quality standards and assess the relevant knowledge, so as to improve the inspection ability. Organize the detailed explanation of the evaluation standard of the learning quality management of the head nurse in the whole hospital and require the head nurse of each department to formulate the improvement plan one by one according to the existing problems in the department, combined with the content of the quality standard, the rectification plan is specifically responsible for by the head nurse, and the whole staff is required to participate. And submit it to the nursing department for approval, and after approval, the head nurse will organize the whole department to carry out the implementation. For the implementation level: hold the quality management-related knowledge training and assessment of the whole hospital, and the assessment items shall be subject to the written examination; the head nurses are required to organize regular scientific meetings to discuss and clarify the quality standards and assessment methods at the scientific meetings. Analyze the errors in the inspection process of the department to find out the existing gap and carry out the division of labor and rectification, and require each department to set up corresponding internal quality control teams, so that everyone has their own responsibility and emphasis, so as to form a good atmosphere for everyone to participate in quality management; nurses should be familiar with their respective management responsibilities and improvement plans for undergraduate problems. Carry on the implementation according to the plan: the implementation process adopts the cycle management mode, that is, the head nurse implements the fixed responsibility cycle management to the nurse, the quality control team leader implements the fixed department cycle management to the head nurse, and the quality improvement leading group implements the fixed item cycle management to the quality control team leader. The head nurse carries out the circular management of responsibility to the nurses, and according to the rectification plan, the head nurse implements the management responsibilities from five aspects: ward management, rescue and treatment materials management, special nursing level basic nursing management, nursing document management and head nurse management to the five responsible persons of the quality control team in the department, and the five responsible persons, respectively, implement the management duties of each nurse according to the Kone group plan. The head of the quality control team shall carry out the cycle management of the department to the head nurse, carry out the relevant inspection to each department according to the standards of each quality control group, and adjust the inspection contents at any time according to the results. The quality improvement leading group implements the fixed cycle management to the quality control team leader, and the quality improvement leading group implements the management responsibilities of five projects, such as ward management, rescue and treatment materials management, special first-level basic nursing management, nursing document management, and head nurse management, to each quality control team leader. (3) Stage C (inspection stage): first self-examination, scientific examination, then quality control group inspection, and finally focus on inspection. Self-examination: nurses should first conduct self-examination according to nursing quality evaluation standards, including daily job responsibilities and management responsibilities, and make standardized records. Scientific investigation: the head nurse made a comprehensive examination once a week according to the evaluation standard of nursing quality. And make standard records and regularly report to the nursing department in the form of accounts. Quality control group inspection: nursing expert supervision group according to the plan to check each clinical department of the hospital once a quarter, key departments once a month. The focus of the inspection is the quality improvement points in the rectification and reform plan of each department, and strive to take the problems existing in the last inspection as the focus of the next inspection. Key check: the nursing expert supervision group takes the common problems and key points and weak links in nursing work as the quality improvement points of the whole hospital to conduct random checks. (4) Stage A (summary and treatment stage) summing up the results of self-examination: nurses are required to report and communicate the results of self-examination in the early shift every day; the head nurse analyzes the evaluation results according to the results of the examination and discusses them at the meeting of science and technology. Timely revision of objectives, improvement measures, and timely follow-up of the progress of the plan and link the results of quality evaluation with the distribution of labor services in the department. The examination results of the nursing expert supervision group were reported at the hospital quality management committee and reported to the whole hospital in the form of OA, the centralized problems were analyzed at the head nurse meeting, and the improvement measures and suggestions were fed back to the relevant clinical departments in time; for the advantages, we should consider how to maintain them in the next cycle. Put forward new problems: the new problems and the common problems existing in the hospital were summarized and put forward by the nursing expert supervision group, which were improved as a continuous quality improvement project, and the standard and plan schedule were revised. The successful experience and shortcomings should be used as the driving force and basis to promote the next PDCA cycle.

### 2.3. Observation Index

#### 2.3.1. Nursing Quality

Nursing quality [7]: the nursing department evaluated the nursing quantity of the two groups from three dimensions (nursing safety, specialist quality, and nursing norms). A total of 12 aspects were assessed twice a month, and 2 points were deducted if a quality defect was found. The nursing quality score was calculated according to 40% nursing safety, 30% specialist quality, and 30% nursing standard. The total score was 100, and the higher the score was, the higher the nursing quality was.

#### 2.3.2. Score of Individual Quality Control Examination in Clinical Department

This research uses the “Evaluation Standard of Nursing quality Control in Clinical Department,” which is being used by the nursing department of this hospital in the assessment of nursing quality in clinical department, as the evaluation index. The evaluation standard is the standard of nursing quality management revised by the members of the joint nursing expert supervision group of the nursing department of the hospital with reference to “Evaluation Indexes of the third-level General Hospital of the Ministry of Health” [8] and ((JCI Certification and quality Hospital Evaluation Index) [9], combined with the actual situation of clinical nursing work. The standard divides the nursing quality management of clinical departments into five dimensions. Among them, the ward management mainly examines the clinical nurses' mastery of basic nursing; the quality management standards of rescue and treatment materials/drugs mainly assess the management of necessary equipment and drugs in the ward; special first-level nursing management mainly evaluates whether nurses can provide timely, safe, and effective holistic nursing for critically ill patients; nursing document management mainly evaluates whether nurses can record the nursing process according to the standards and norms. The management of head nurses is mainly comprehensive supervision and inspection. The higher the score, the better the effect of individual quality control examination in clinical department.

#### 2.3.3. Nursing Quality Score in Operating Room

Nursing quality score of the operating room [10]: one day after the operation, the head nurse regularly scored the nursing quality of the whole operation process, including equipment management, equipment preparation, nurses' cooperation skills, disinfection and isolation quality, and the total score. The full score is 100, and the higher the score, the better the nursing quality in the operating room.

#### 2.3.4. Incidence of Adverse Events and Nursing Errors in Operation

Statistics of the incidence of adverse events and nursing errors between the two groups, including nosocomial infection, iatrogenic injury, information check errors, equipment failures, violation of operation regulations, ECG monitoring errors, infusion operation errors, and medication errors.

#### 2.3.5. The Number of Problems Existing in the Quality Management of Nursing Documents

Statistics were made on the number of problems existing in the quality management of nursing documents in the two groups, including temperature sheets, medical orders, evaluation sheets, nursing records, and other nursing documents.

#### 2.3.6. Satisfaction Score

Evaluation of patient satisfaction [11]: the patient satisfaction questionnaire was used to evaluate the patient satisfaction of the two groups. The questionnaire included 10 items and 5 dimensions (nursing communication, professional technology, nursing service attitude, nursing environment, and knowledge education). The total score was 20-100, and the higher the score was, the higher the patient satisfaction was.

### 2.4. Statistical Analysis

Using SPSS21.0 statistical software, before statistical analysis, the measurement data were tested by normal distribution and variance homogeneity analysis to meet the requirements of normal distribution or approximate normal distribution, expressed as $\bar{x}\pm s$, and repeated measurement data were analyzed by repeated measurement analysis of variance. *T*-test was used to compare the two groups, *n* (%) was to represent the counting data, and *χ*^2^ test was used. The difference was statistically significant when *P* < 0.05.

## 3. Results

### 3.1. Comparison of Nursing Quality

Compared to the control, in the comparison of nursing quality, the nursing safety, specialty quality, and nursing norms in the study group were higher (*P* < 0.05). All the results are presented in Figure 1.

### 3.2. Comparison of Individual Quality Control Examination Scores in Clinical Departments

Compared to the control, in terms of the scores of individual quality control examination in clinical departments, the scores of ward management, rescue, therapeutic articles, drug management, first-level nursing, nursing documents, and head nurses in the study group were higher (*P* < 0.05). All the results are illustrated in Table 1.

### 3.3. Comparison of Nursing Quality Score in Operating Room

Compared to the control, in terms of the operating room nursing quality score, the instrument management, instrument preparation, nurses' cooperation skills, disinfection and isolation quality, and the total score were higher in the study group (*P* < 0.05). All the results are shown in Table 2.

### 3.4. Comparison of the Incidence of Adverse Events and Nursing Errors in Operation

Compared to the control, in terms of the incidence of operative adverse events and nursing errors, the incidence of nosocomial infection, iatrogenic injury, information check error, equipment failure, violation of operation regulations, ECG monitoring error, infusion operation error, and medication error in the study group was lower (*P* < 0.05). All the results are illustrated in Table 3.

### 3.5. Comparison of the Number of Problems Existing in the Quality Management of Nursing Documents

According to the comparison of the number of problems existing in the quality management of nursing documents, compared with the control, the number of problems in temperature sheet, medical order, evaluation sheet, nursing record, and other nursing documents in the study group was lower (*P* < 0.05). All the results are illustrated in Table 4.

### 3.6. Comparison of Satisfaction Score

Compared to control, the scores of nursing communication, professional technology, nursing service attitude, nursing environment, and knowledge education in the study group were higher (*P* < 0.05). All the results are shown in Table 5.

## 4. Discussion

With the advancement of the traditional medical model and the implementation of the new medical reform, the requirements of the society and patients for the medical quality and nursing service quality of the hospital are increasing, which renders the nursing management, especially the nursing quality management, become particularly important [12, 13]. Nursing quality is the overall embodiment of nursing theoretical knowledge, technical level, working attitude, and nursing effect of nursing staff, which is the core content of nursing management and closely linked to the health and life of patients [13]. The quality of nursing directly affects the overall medical quality of the hospital. Therefore, to survey how to improve and enhance the quality of nursing has become the primary task of hospital nursing work [14]. Nursing quality management is a comprehensive management measure to make the nursing quality reach the best standard under the condition of certain human, financial, and material resources. Meanwhile, it is also an important management measure to improve nursing skills and improve the image of nurses [15]. In the new situation, nursing quality management can meet the demand of modern medicine only if it develops in a standardized, systematic, and scientific direction. Since the 1990s, with the exchange and cooperation of nursing experience at home and abroad, nursing management in China has become one of the important contents of medical and health reform [16]. In recent years, China has made some progress in nursing theoretical research and practical research. More and more managers and nursing workers apply modern management theory to nursing quality management and put it into practice, demonstrating the mode of nursing quality management has been continuously improved [17]. PDCA cycle theory has become one of the successful and effective management models for nursing managers.

PDCA cycle was put forward by Dr. Deming, an American quality management expert in the 1950s. Its main content is the abbreviation of plan, do, check, and action. It is the basic tool of total quality management [18]. The PDCA cycle can be divided into 4 stages: 1 planning stage, 2 implementation stage, 3 inspection stage, and 4 treatment stage. These four stages can often be carried out successively or at the same time. In the actual work, the specific operation is first set work objectives or ask questions, and then through the analysis of the problems, find out the induces of the problems, then formulate corresponding measures, and implement measures. In the process of implementation, through the evaluation of the effectiveness of the implementation, sum up the experience, and move on to the next cycle. It is an example of an effective management method that is constantly improving and spiraling up. The ultimate goal of management is to optimize all kinds of work [19, 20]. The PDCA cycle mode accords with the objective law of “practice, cognition, and re-practice cognition” and embodies the scientific epistemology. Therefore, the PDCA cycle is regarded as a universal and practical management philosophy [21]. This standardized and scientific management procedure was first applied to enterprise management and achieved good results [22]. Considering its rigorous operating procedures and diverse management levels, PDCA cycle is suitable for different kinds of management, which is regarded as an effective method to strengthen internal management by various industries at home and abroad, and it is also suitable for all aspects of management work and management [23–25].

In view of the results of our current study, the nursing quality, nursing safety, specialty quality, and nursing norms were higher in the study group. With regard to the scores of individual quality control examination, the scores of ward management, rescue, therapeutic articles, drug management, first-level nursing, nursing documents, and head nurses were higher in the study group. According to the comparison of the number of problems existing in the quality management of nursing documents, the number of problems in temperature sheet, medical order, evaluation sheet, nursing record, and other nursing documents was lower in the study group. The writing of nursing records not only reflects the dynamic changes of patients' medical and nursing process and condition during hospitalization but also is the basis for evaluating the professional ability of nurses and nursing quality management. In this study, the problems of nursing documents mainly exist in temperature sheet, doctor's order, evaluation sheet, and nursing record. Through comprehensive analysis, nurses' lack of understanding of the rigor and importance of nursing records, heavy burden on nursing staff, and untimely quality control of nursing records is the main reason for the nonstandard writing of nursing records [26, 27]. Through the conduction of PDCA cycle, the work quality of nurses was effectively improved, and the problems of nursing documents were further reduced.

In this study, the scores of nursing quality in operating room, equipment management, equipment preparation, nurses' cooperation skills, disinfection and isolation quality, and total score were higher in the study group. With regard to the incidence of operative adverse events and nursing errors, the incidence of nosocomial infection, iatrogenic injury, information check error, equipment failure, violation of operation regulations, ECG monitoring error, infusion operation error, and medication error was lower in the study group. The scores of nursing communication, professional technology, nursing service attitude, nursing environment, and knowledge education in the study group were higher than those in the control group. The possible reason for our results is that in the past, nursing quality management has been dominated by experience management, that is, “housekeeping” or “paternalistic” management mode, which is lack of science and effectiveness and lack of guarantee for nursing quality [28]. In recent years, more nursing workers and managers apply modern management theory to nursing quality management and put it into practice. Nursing quality management model is constantly improved [29]. PDCA cycle theory is one of the successful and effective management models for nursing workers. The PDCA cycle is divided into 4 stages: planning stage, implementation stage, inspection stage, and treatment stage. These four stages are often carried out at the same time. Advantages of PDCA cycle that the big ring covers the small ring and advances layer by layer can greatly enhance the execution efficiency of the work, which further improves the nursing quality of the day operation ward [30].

Taken together, the adoption of PDCA process management can effectively enhance the nursing quality and safety of the day operation ward, further improve the quality of hospital nursing work, and elevate patient satisfaction. This new nursing model based on PDCA will exert great potential and application value in the management of day ward in the future.

## Figures and Tables

**Figure 1:** Comparison of nursing quality between the two groups.

**Table 1:** Comparison of individual quality control scores between two groups of clinical departments ($\bar{x}\pm s$, points).

Group	*N*	Ward management	Rescue and therapeutic articles	Drug management	Special nursing first-class nursing	Nursing documents	Head nurse management
Control group	20	85.96 ± 2.50	84.95 ± 1.22	85.93 ± 2.11	86.83 ± 1.25	86.84 ± 2.11	86.94 ± 1.45
Research group	20	92.85 ± 1.93	94.82 ± 1.22	91.85 ± 2.34	95.39 ± 1.29	94.84 ± 1.22	94.82 ± 1.22
*t*		9.756	25.583	8.402	21.311	14.678	18.596
*P*		<0.01	<0.01	<0.01	<0.01	<0.01	<0.01

**Table 2:** Comparison of nursing quality score in operating room ($\bar{x}\pm s$, points).

Group	*N*	Instrument and equipment management	Equipment preparation	Nurses' cooperation skills	Disinfection and isolation quality	Total score
Control group	20	23.95 ± 2.11	15.96 ± 2.14	24.85 ± 2.53	15.92 ± 1.24	84.85 ± 1.45
Research group	20	26.94 ± 2.05	18.93 ± 1.22	28.93 ± 1.56	19.93 ± 2.11	94.95 ± 2.93
*t*		4.545	5.391	6.138	7.327	13.816
*P*		<0.01	<0.01	<0.01	<0.01	<0.01

**Table 3:** Comparison of the incidence of adverse events and nursing errors between the two groups ($\bar{x}\pm s$, points).

Group	*N*	Nosocomial infection	Iatrogenic injury	Information checking error	Out of order	Violate the operating regulations	ECG monitoring error	Error in infusion operation	Medication error	Total incidence rate
C	20	1 (5.00)	2 (10.00)	3 (15.00)	1 (5.00)	1 (5.00)	1 (5.00)	1 (5.00)	1 (5.00)	11 (55.00)
R	20	0	0	0	1 (5.00)	0	1 (5.00)	0	0	2 (10.00)
*X* ^2^										9.230
*P*										<0.01

**Table 4:** Comparison of the number of problems in the quality management of nursing documents between the two groups of nurses (*n*/%).

Group	Cases	Temperature sheet	Doctor's order	Evaluation form	Nursing record sheet	Other
Control group	20	6 (30.00)	6 (30.00)	7 (35.00)	6 (30.00)	9 (45.00)
Research group	20	1 (5.00)	1 (5.00)	0	0	0
*X* ^2^		4.320	4.320	8.484	7.058	11.612
*P*		0.037	0.037	<0.01	<0.01	<0.01

**Table 5:** Comparison of patient satisfaction scores ($\bar{x}\pm s$, points).

Group	*N*	Nursing communication	Professional technology	Nursing attitude	Nursing environment	Knowledge education
Control	80	15.96 ± 2.91	15.92 ± 1.29	14.95 ± 2.91	16.83 ± 1.22	15.93 ± 1.21
Research	80	19.92 ± 0.43	19.82 ± 0.21	18.85 ± 0.53	19.85 ± 0.53	19.72 ± 0.34
*t*		6.020	13.344	5.896	10.153	13.485
*P*		<0.01	<0.01	<0.01	<0.01	<0.01

## Data Availability

No data were used to support this study.

## References

[1] Qingjun G., Xiuping L., Zhixia F. (2021). The influence of PDCA continuous quality improvement management on the efficiency of equipment management in operating room. *Management of Health Standards in China*.

[2] Huixia C., Fang J. (2022). Investigation on knowledge, belief and practice of PDCA circulation management intervention on prevention of deep venous thrombosis among nurses in operating room. *Thrombus and Hemostasis*.

[3] Yongmei S. (2021). Application effect and pain degree analysis of operating room nursing based on PDCA mode in senile elective orthopedic surgery. *Contemporary Journal of Clinical Medicine*.

[4] Jiang L., Sun X., Ji C., Kabene S. M., Keir M. Y. (2021). PDCA cycle theory based avoidance of nursing staff intravenous drug bacterial infection using degree quantitative evaluation model. *Results in Physics*.

[5] Gu S., Zhang A., Huo G. (2021). Application of PDCA cycle management for postgraduate medical students during the COVID-19 pandemic. *BMC Medical Education*.

[6] Kong X., Zhu X., Zhang Y., Wu J. (2021). The application of plan, do, check, act (PDCA) quality management in reducing nosocomial infections in endoscopy rooms: it does work. *International Journal of Clinical Practice*.

[7] Lyu J., Wang K., Liu J., Wang X., Zhang C. (2021). The innovative application of PDCA cycle mode in the cost control of drilling and completion in Caofeidian area of Bohai oilfield. *Journal of Innovation and Social Science Research*.

[8] Chigeng Z., Zhipeng J., Shen B. (2021). Research on flipped classroom teaching based on OBE and PDCA—take Jiaxing vocational and technical college’s “virtual reality interactive design foundation” course as an example. *Vocational Education*.

[9] Tang B., Lin D., Zhang F., Yan M., Shao A. (2021). The “plan-do-check-action” plan helps improve the quality of the “standardized training of resident physicians”: an analysis of the results of the first pass rate. *Frontiers in Public Health*.

[10] Jianming L. (2021). Research on the mode of innovative talent cultivation in the multi-synergy integrated circuit industry based on the PDCA cycle theory. *Journal of Physics: Conference Series*.

[11] Zhou J., Xu H., Jiang M. (2021). Effect of PDCA-based nursing management model on the quality of life and complications of patients with acute leukemia undergoing chemotherapy. *American Journal of Translational Research*.

[12] Huang L., Lu C., Pang M. (2021). Effect of PDCA-based nursing intervention on activities of daily living, neurological function and self-management in acute cerebral stroke. *American Journal of Translational Research*.

[13] Leitmann A., Reinert S., Weise H. (2020). Surgical suture course for dental students with the Peyton-4-step approach versus the PDCA cycle using video assisted self-monitoring. *BMC Oral Health*.

[14] Xu X., Qian X., Lv X. (2019). Application of FOCUS-PDCA in reproductive clinic procedure and study on patient satisfaction. *Indian Journal of Pharmaceutical Sciences*.

[15] Wei Y., Xu M., Wang W. (2020). Effect analysis of PDCA cycle method applied in nursing management of disinfection supply room. *Panminerva Medica*.

[16] Chen Y., Zheng J., Wu D., Zhang Y., Lin Y. (2020). Application of the PDCA cycle for standardized nursing management in a COVID-19 intensive care unit. *Annals of Palliative Medicine*.

[17] Li Y., Wang H., Jiao J. (2020). The application of strong matrix management and PDCA cycle in the management of severe COVID-19 patients. *Critical Care*.

[18] Sunadi S., Purba H. H., Hasibuan S. (2020). Implementation of statistical process control through PDCA cycle to improve potential capability index of drop impact resistance: a case study at aluminum beverage and beer cans manufacturing industry in Indonesia. *Quality Innovation Prosperity*.

[19] Peng W. (2019). Application of PDCA cycle based on "blue ink cloud class" in learning management of secondary vocational nursing internship. *Journal of Network Computing and Applications*.

[20] Qiu Y.-X., Zhao C.-Y., Zhu J.-M., Li L.-J. (2019). Analysis of the application and practice of PDCA cycle in management of the naked medicine dispensing—the quality and safety of the drug. *Frontiers of Nursing*.

[21] Wang Q., Ma J., Yan M., Yan Y., Wang Y., Bian D. (2019). The effect of PDCA cycle management method on the promotion of nursing quality management in the operating room. *American Journal of Nursing Science*.

[22] Jie X., Guoqin R., Chun B. (2019). Application of PDCA circulation in improving the execution rate of preoperative time out based on JCI standard. *Nursing Research*.

[23] Xuemei L. (2019). Application of PDCA circulation management in restlessness nursing of patients in recovery period of anesthesia. *Nursing Science*.

[24] Huihua S., Liying Y., Mengjiao X. (2018). Using FOCUS-PDCA program to reduce the incidence of sterilized wet bags of foreign medical devices. *Nursing Research*.

[25] Tianying D., Min Z. (2017). Practice and application of quality control circle in nursing quality management in operating room of trauma center. *PLA Journal of Nursing*.

[26] Tianying D., Min Z. (2017). Practice and application of quality control circle in nursing quality management in operating room of trauma center. *PLA Journal of Nursing*.

[27] Qian W., Jie M., Yaling Y. (2017). PDCA cycle management method improves doctors' satisfaction with the cooperation of nurses in operating room. *PLA Journal of Nursing*.

[28] Liang C., Xia L., Yiqin Z. (2017). PDCA management of network sharing of general package electronic atlas in central supply room. *Journal of Nursing*.

[29] Li Hong Y., Xiaohua (2016). Application of PDCA in clinical nursing teaching in operating room. *Chongqing Medicine*.

[30] Yongfeng C. (2015). Application effect of PDCA circulation in nursing safety management in operating room. *PLA Journal of Nursing*.

